The article "New Quality Cost Framework (QCF) Based on the Hybrid Fuzzy MCDM Approach" was published in 2022. Journal: Comput Intell Neurosci.

# New Quality Cost Framework (QCF) Based on the Hybrid Fuzzy MCDM Approach

**DOI:** 10.1155/2022/6416989

**Published:** 2022-03-28

**Authors:** Qiong Wu, Jing Xuan, Fuli Zhou, Yuanfei Mei, Jiafu Su

**Affiliations:** ^1^College of Management Science and Engineering, Chongqing Technology and Business University, Chongqing 400067, China; ^2^Chongqing Research Center for Industrialization and Informatization Integration and Logistics Information Technology Application, Chongqing, China; ^3^Postdoctoral Research station of Changzufeiyue (CZFY) Technology Development Co., Ltd, Chongqing 402360, China; ^4^College of Language Intelligence, Sichuan International Studies University, Chongqing 400067, China; ^5^College of Economics and Management, Zhengzhou University of Light Industry, Zhengzhou 450001, China; ^6^International College, Krirk University, Bangkok 10220, Thailand

## Abstract

Quality cost framework (QCF), as a measurement tool and research method, has played a significant role on quality improvement procedure (QIP) and recognition on economics of quality. The four general QCFs are usually conceptually employed assist quality managers to measure the quality cost (QC/COQ) including PAF, intangible loss, process cost, and ABC framework. The question of how to select an appropriate quality cost framework for individual organization is of great significance for implementing quality improvement activities. Considering the *effectiveness* and *feasibility* of the alternative solution, a novel hybrid fuzzy MCDM approach integrating fuzzy DMEATEL, an antientropy weighting technique and FVIKOR method are employed to study the quality cost models and assist managers to select a best QCF for an auto factory. The combined weight from subjectivity and objectivity is embedded into fuzzy VIKOR procedure to obtain alternatives' ranking order. The case study in a Chinese automaker enterprise shows high robustness of the hybrid MCDM approach, and it assists quality mangers to perform quality cost practice. Different from the previous study, the preferred solution is the ABC quality cost framework when feasibility dimension dominates, while the intangible loss framework shows first priority when the organization focuses on effectiveness principle.

## 1. Introduction

With an increasing fierce marketing situation and multiple products in the auto industry, quality was treated as a crucial element and core competence for industrial organizations [1, 2]. Auto-makers began to focus on quality improvement programs and customer satisfactions' enhancement by quality tools such as total quality management (TQM), lean six sigma (LSS), 8D, and statistical process control (SPC) technique [3–8]. However, with continuous quality improvement practice (QIP), managers in self-brand auto firms show their interests on economics of quality improvement activities. Quality management (QM) practice, for instance, supplier quality factor, processing technology, and procedure control have proven to be an effective method to promote quality performance [9]. As all industries exist, quality does not come for free as it bears extra inputs and investment. While there are few relative cost measurements during QM practice, especially for expenditures of the quality improvement program (QIP) in self-brand automotive firms. Besides, quality costing becomes an effective trigger and method to control quality improvement activities in the automobile industry [10].

The purpose of QIP is to improve the product performance with lower cost [11] to meet the requirement of customers, which stimulates the cost of quality model development [12–14]. Freiesleben targeted profit maximization as the objective by taking quality investment, cost of poor quality and revenue effect of better quality into account instead of the cost minimization objective [15]. While the prerequisite work of all these quality innovations is the total quality related cost measurement, to collect quality costs an organization needs to adopt a framework to classify costs. Therefore, it is of great significance and urgency for managers to choose an appropriate quality cost framework (QCF) to recognize the economics of quality [11, 16].

Quality cost (QC) has proven to be an effective way for quality improvement and cost reduction. The concept of quality cost (QC), first proposed by Juran and Feigenbaum, has been studied and applied as an effective tool for cost reduction and quality improvement [11, 17]. Similar to the definition of lifecycle cost (LCC), the COQ focuses on the quality-related cost from product lifecycle perspective [18]. Cost of quality (COQ) represents the cost of not achieving good quality. Any expenditure due to substandard quality contributes to the cost of quality. The term is referred to as “quality related cost,” “poor quality cost”, or “cost of poor quality,” all of which focus on the failure expenditure when the quality cannot meet the customer. Based on the definition of American Society for Quality Control (ASQC, 1971), cost of quality is a methodology that allows an organization to determine the extent to which its resources are used for activities that prevent poor quality that appraise the quality of the organization's products or services, and that result from internal and external failures [19–21].

Quality cost framework and accounting systems are part of every modern organization's quality improvement strategy, and help management plan for quality improvement by identifying opportunities for a greatest return on investment. While there is no general agreement on the definition of COQ, and the specific quality cost differs from author to author, as well as for different industry and organization. As quality scholars and experts advocate that quality cost framework should be tailor-made for particular industrial organization [16]. In order to identify the quality cost items, some organizations are trying to develop its quality cost system based on the quality cost framework (QCF) linking with its own financial accounting system. The cost items can be calculated based its specific activity and cost parameters. The quality cost program is a systematic task whose items need to be developed, modified, deleted, and adjusted according to quality improvement practice and the practical situation of the organization.

Because there are many conceptual quality cost frameworks can guide the organization to develop its COQ program, the appropriate QCF is the crucial step for its success. Moreover, it is important for different individual organizations to choose the most appropriate quality cost framework for better quality management practice. Because the quality cost framework selection is a complicated research problem subjecting to multiple criteria of the individual organization. The quality cost framework selection can be regarded as a multicriteria decision-making problem with respect to multiple conflicting criteria. The MCDM theoretical models have been regarded as truimple for dealing with the comprehensive evaluation of industrial problems with multiple conflicting criteria [22]. Tsai initially explored a hybrid DEMTELA-ANP model to deal with this issue [16]. However, decision-making techniques are subjectivity-oriented, and it is difficult to collect the decision information with crisp value for the Chinese auto factories [23, 24]. Due to lack of researches in terms of quality innovation on QCF selection, this paper aims at assisting managers to evaluate and select the best quality cost framework to fill the gap by a hybrid fuzzy multi-criteria decision-making (MCDM) method considering the effectiveness and feasibility of alternative model. Meanwhile, the fuzzy-based method has been employed to deal with the uncertainty and vagueness of decision information which facilitates to the data collection for decision makers. This paper aims to enhance the capacity of auto factories to prioritize quality cost framework by a hybrid MCDM approach and address the quality cost innovation. The main contributions of this paper are as follows. First, the hybrid fuzzy multi-criteria decision-making approach integrating fuzzy DEMATEL, anti-entropy weighting technique and VIKOR method is employed for QCF selection, which facilitates data collection and easy implementation. Second, the seven criteria from effectiveness and feasibility of quality cost framework are addressed based on the barriers in COQ model, and the criteria relationship map (CRM) is illustrated in the two-dimension clusters. Third, the combined weighting technique from subjectivity and objectivity has been embedded into fuzzy VIKOR procedure, which makes the approach more flexible according to the decision makers' preference.

The rest of this paper is structured as follows.  Section 2 provides the literature review on quality cost related topics. The hybrid MCDM approach integrating fuzzy DEMATEL, anti-entropy weighting technique, and fuzzy VIKOR method is employed to deal with the QCF selection in the next section. In Section 4, a case application is presented in a self-brand auto-factory and this paper is ended with conclusions in Section 5.

## 2. Literature Review

### 2.1. Development and Application of QCFs

The quality cost has experienced several decades by researchers and practitioner from all walks of life [21, 25–33], while the concept for different organization or industry has been argued by many researches, due to different considerations and specific procedures. The broad concept of “economics of quality” and “cost of quality” can be traced back to the early 1950s [33]. After the initial researches by Feigenbaum (1956), Juran (1951), and Crosby's (1979) etc., the basic philosophy of quality cost has been widely used and studied with high agreement and appreciation [34]. The prevailing four quality cost frameworks applied in the quality practice are prevention-appraisal-failure (PAF), the intangible loss framework, process cost framework and activity-based cost (ABC) [11, 16, 33, 34] are presented in Table 1.

The quality cost concept, first proposed in Juran's “quality control handbook” and in Feigenbaum's “total quality control” [33]. The specific PAF framework is propounded and has been adopted by many researchers and practitioners. There are three categories in this cost framework including prevention cost, appraisal cost, and failure cost. Prevention cost consists of cost items are associated with activities launched to prevent poor quality in products or services. Appraisal costs are related to measurement, evaluation, or auditing products or service to guarantee conformance to quality specification and performance requirements. Failure cost includes cost items leading to products or services not conforming to customer needs from the defective's standpoint, and it can be divided into internal and external failure cost. The PAF cost framework, as a prevailing COQ model, has been applied into many industries for quality costing [31, 32, 48–50], and it is also employed to optimize the quality cost and obtain the optimal quality level [13, 40, 51–53].

With the concentration of customers' satisfaction, loyalty, and brand reputation, the intangible loss cost framework has been recently emphasized by extending the PAF model. Actually, in this group of models' intangible loss or opportunity loss cost is incorporated into a typical P-A-F model, which contained the revenue lost and profit not earned due to the customer complaints. Wang owed customer satisfaction and complaint after-sales to the intangible loss and the traditional COQ models has been illustrated [34]. Snieska et al. divided the hidden costs that are always neglected and usually hardly measured caused by failed quality, into three elements: customers' goodwill, brand value, and image of company [41]. As the quality cost measurement is a systematic work which need multidepartment involvement, Yang redefined the “extra resultant cost” and “estimated hidden cost” on the basis of traditional PAF COQ model, which can be measured by quality cost account matrix and responsible weight of each department [45]. Liapis et al. studied intangible quality related cost in fuel supply chain including quality deficits, customer complaint, product mixtures, and negative impacts, etc. [46]. Palikhe studied the detailed quality cost construction considering opportunity cost in electric utility industry based on the PAF framework [54]. This group of models emphasizes the role of intangible cost within the overall quality cost scheme and focuses on the hidden loss, which helps quality managers to recognize the economics of quality and its products' performance better.

In view of a number of drawbacks of the PAF cost framework, the process cost framework developed by Crosby concentrated on the operation process rather than the products or services. The process cost framework has two segments that are cost of conformance (COC) and cost of un-conformance (CONC), and the quality term is treated as “conformance to customers' requirements.” The conformance cost is the cost involved in making certain things are performed right at the first time, which is similar to actual prevention and appraisal costs, while the un-conformance cost is the expenditure wasted when the work fails to conform to customer requirements, calculated by recognizing the cost of reworking, correcting, scrapping activities, which is similar to failure cost. Daunorienė has studied the COQ model from the value added chain perspective, which provided an effective way to evaluate the quality cost of the value added chain's procedures [47]. Teli et al. has proven quality cost technique to be a significant tool to reduce total costs in the automobile industry without compromising quality, which presents a case study on failure cost analysis based on Crosby philosophy [50]. The cost items need to be measured based on specific processes and it is influenced by the conformance level. The application of process cost framework is suggested as a preferred method for quality costing under TQM environment due to its quick response on quality issues [34], and it helps quality mangers to identify the importance of process cost measurement and ownership with a more integrated framework [33, 55]. Understanding the related process sufficiently is the first step in quality costing program based on process cost framework; however, the complete concise activity analysis linked with specific process without duplication for an organization may be time-consuming compared with PAF framework.

Even though the above three quality cost frameworks provide management insight on quality costing based on the economics of quality; however, it still cannot provide appropriate methods to include overhead cost items. In other words, the three frameworks are effective enough to cover the cost items and reflect the quality actions in the continuous quality improvement procedure (CQIP), while all of them are category philosophy lacking of feasibility and specific calculation on overhead costs. In addition, due to the lack of quality related data and un-conformance of traditional accounting system, the three frameworks fail to measure the quality improvement benefits, as well as cost elements. Activity-based costing method, first developed by Cooper and Kaplan, filled this gap and was adopted to identify and assign every cost activity to products and services in an organization. It assigns more overhead expenditures into dire costs and is more compatible with cost measurement system. Jorgenson and Enkerlin [56] presented a quality cost program based on ABC framework to identify, quantify, and allocate cost by a manufacturing organization. The ABC method is an alternative way that can recognize the cost items, instead of a COQ model. Based on the activity-oriented cost (ABC) framework, it is preferred for the auto factory to eliminate the nonvalue-added activities and invest much more effectively during its quality improvement procedure (QIP).

The abovementioned four quality cost frameworks have been widely used by experts and quality practitioners. In addition, some of the above cost frameworks have proven to be adopted by many standard organizations as presented in Table 2.

### 2.2. Criteria for QCF Selection

Even though the quality cost framework provides an effective guidance on quality costing, there are many barriers for the quality cost practice due to the lack of quality related data and limited cost information, etc. It is a prevailing phenomenon that many departments usually ignore the importance of the quality cost reporting in Chinese auto factories. The quality manager always focuses quality improvement procedures and quality indexes such as failure frequency (R/1000). Customer complaints and things go wrong (TGW) indicator, ignoring economics of quality [20, 50]. Due to the difficulty on the benefit measurement and invisibility of the immediate improvement, financial manager does not show much interest on quality cost reporting. The less involvement and lack of management support or absence of management interests are the barriers in tracking such costs [20]. In addition, due to the lack of knowledge and cost un-conformance with traditional accounting system, the organization cannot perform quality costing program based on an appropriate quality cost framework (QCF). The well-organized data structure and multi-department involvement based on the appropriate quality cost framework can resolve the dilemma, which helps manager to identify the cost elements and data collection with higher efficiency. Therefore, an appropriate QCF is the crucial step for organizations. Based on previous studies [16, 38, 57, 58], seven criteria from two dimensions are categorized (illustrated in Table 3) to implement this research.

To recognize the most suitable quality cost framework for an organization, a hybrid fuzzy decision-making framework is employed to deal with this problem based on the established criteria hierarchy.

## 3. Fuzzy Hybrid MCDM Approach for QCF Selection

The purpose of this research is to select the most appropriate quality cost framework for an automotive organization with integrated fuzzy DEMATEL-AEW-FVIKOR approach. The quality cost framework selection is regarded as a *MCDM* problem subject to criteria set *C*={*C*_1_, *C*_2_,…, *C*_*j*_,…, *C*_*n*_}, which includes decision makers *DM*={*DM*_1_, *DM*_2_,…, *DM*_*k*_,…, *DM*_*K*_} and alternative set *A*={*A*_1_, *A*_2_,…, *A*_*i*_,…, *A*_*m*_}. Suppose ${\tilde{x}}_{kij}$ is the rating of *i*-th alternative with respect to *j*-th criterion provided by the *k*-th representative, which is represented by the triangular fuzzy number converted from linguistic terms. In addition, the criteria combined weight has been divided into subjective and objective aspect. Let the relative subjective weight is presented as **w**^*s*^=(*w*_1_^*s*^, *w*_2_^*s*^,…, *w*_*j*_^*s*^,…*w*_*n*_^*s*^), and the objective weight of criteria is **w**^*o*^=(*w*_1_^*o*^, *w*_2_^*o*^,…, *w*_*j*_^*o*^,…, *w*_*n*_^*o*^). The *φ* index is the relative importance of subjective item, and the criteria combined weight is **w**^*c*^=(*w*_1_^*c*^, *w*_2_^*c*^, *w*_*j*_^*c*^,…, *w*_*n*_^*c*^) integrated with the subjectivity and objectivity. In order to figure out the cause and effect relationship among the criteria, every expert is asked to make a comparison with the direct effect of criterion *C*_*i*_ on criterion *C*_*j*_ with linguistic variables. There are five levels to express the influence degree (Table 4) and let ${\tilde{p}}_{kij}$ is the influence degree rating of criteria *C*_*i*_ on criteria *C*_*j*_ provided by the *k*-th expert [59].

### 3.1. Fuzzy-Based Techniques

Linguistic variable has been utilized for the multicriteria decision-making problem for the uncertainty and vagueness of the decision information [62, 63]. It helps to collect decision information provided by investigated representatives and can transform the linguistic description into mathematical information. The fuzzy set, introduced by Zadeh in 1965, is an effective tool to deal with the uncertainty and ambiguity of human judgment and evaluation in decision-making science [60]. In practice, it is difficult to recognize the crisp numbered information of the investigated alternatives, which motivates the application of fuzzy-based techniques [64, 65]. It is much better to convert linguistic terms into qualitative fuzzy numbers [66, 67]. The triangular fuzzy number (TFN) has been adopted to quantify the corresponding linguistic term [68].

#### 3.1.1. Triangular Fuzzy Number and Linguistic Variable

**Definition 1 (Fuzzy set).**

Let *X* be the universe of discourse, and. the fuzzy set *A* can be regarded as order pairs, which are linked by a membership function that maps each element with the number. The function value is the membership degree for *x*. The fuzzy number is a particular case of a fuzzy set, which is used to represent the vague scale ratings of the objective.

**Definition 2 .**

According to the shape of membership function, the fuzzy numbers can be divided into several forms. Assume triangular fuzzy number $\tilde{A}$ = (*a*, *b*, *c*) and its membership function can be illustrated as Figure 1 shows.

(1) $$\begin{array}{c} \mu_{\bar{A}}\left(x\right)=\left\{\begin{array}{cc} \frac{\left(x-a\right)}{\left(b-a\right)}, & a\leq x\leq b,\\ \frac{\left(c-x\right)}{\left(c-b\right)}, & b\leq x\leq c.\\ 0, & \text{otherwise} \end{array}\right.. \end{array}$$

There are two kinds of linguistic terms that need to be defined for the measurement of criteria influence description (Table 4) and rating scales of four quality cost frameworks with respect to each criterion (Table 5). Linguistic variables and corresponding rating scales with TFNs are presented in the following two tables.

#### 3.1.2. Fuzzy Operators and Defuzzification Method

Assume there are two triangular fuzzy numbers *A*_1_=(*a*_1_, *b*_1_, *c*_1_) and *A*_2_=(*a*_2_, *b*_2_, *c*_2_), the algebraic operations are implemented according to the fuzzy operators “⊖” [70]. The common operations between these TFNs can be formulated as follows.

Addition operator: *A*_1_⊖*A*_2_=(*a*_1_+*a*_2_, *b*_1_+*b*_2_, *c*_1_+*c*_2_)

Subtraction operator: *A*_1_⊖*A*_2_=(*a*_1_ − *a*_2_, *b*_1_ − *b*_2_, *c*_1_ − *c*_2_)

In addition,

(2) $$\begin{array}{c} \lambda A_{1}=\left\{\begin{array}{cc} \left(\lambda a_{1},\lambda b_{1},\lambda c_{1}\right), & \lambda \geq 0,\;\lambda \in R\\ \left(\lambda c_{1},\lambda b_{1},\lambda a_{1}\right), & \lambda <0,\;\lambda \in R. \end{array}\right. \end{array}$$

Through the abovementioned fuzzy operators, we can aggregate decision information provided by expert panels. The decision information aggregation can be formed based on the following equation:

(3) $$\begin{array}{c} {\tilde{x}}_{ij}=\frac{\left({\tilde{x}}_{ij}^{1}⊕{\tilde{x}}_{ij}^{2}⊕\ldots ⊕{\tilde{x}}_{ij}^{k}⊕\ldots ⊕{\tilde{x}}_{ij}^{K}\right)}{K}. \end{array}$$

Fuzzy numbers usually require to be transferred into crisp value for ranking and prioritization purpose, whose process called defuzzification. The GMIR method was employed to transfer the TFNs into crisp values as equation (4) shows [71].

(4) $$\begin{array}{c} x_{ij}=\text{defuzzy}\left({\tilde{x}}_{ij}\right)=\frac{x_{ij}^{L}+4x_{ij}^{M}+x_{ij}^{U}}{6}. \end{array}$$

### 3.2. Subjective Weight with the Fuzzy DEMATEL Method

The decision-making and trial evaluation laboratory (DEMATEL) method, first proposed in 1976, has been used to visualize the structure of complicated casual interactions. It helps decision makers to recognize and portray the causes and effects of the criteria with a diagraph map [59]. It has proven to be a big challenge for decision makers to provide crisp values of influence degree of the criteria. In that case, fuzzy logic has been embedded called fuzzy DEMATEL technique has been applied into the subjectivity weight study to address the uncertainty, vagueness, and information leaks. Implementation procedures of the fuzzy DEMATEL method are as follows [72]:

Step 1: Initial direct influence average fuzzy matrix $\tilde{P}$ construction
Based on the linguistic term and corresponding TFNs, the direct influence degree ${\tilde{p}}_{kij}=\left(p_{ijk}^{L},p_{ijk}^{M},p_{ijk}^{U}\right)$ can be converted that *C*_*i*_ on *C*_*j*_ by expert *k*. The diagonal element values of matrix *P* should be zero based on the definition of influence degree. After the fuzzy aggregation through fuzzy operators, the elements ${\tilde{p}}_{ij}=\left(p_{ij}^{L},p_{ij}^{M},p_{ij}^{U}\right)$ in the initial direct influence average fuzzy matrix $\tilde{P}$ can be generated as follows:
  (5) $$\begin{array}{c} {\tilde{p}}_{ij}^{L}=\frac{1}{K}\overset{K}{\underset{k=1}{\sum }}p_{kij}^{L},\\ {\tilde{p}}_{ij}^{M}=\frac{1}{K}\overset{K}{\underset{k=1}{\sum }}p_{kij}^{M},\\ {\tilde{p}}_{ij}^{U}=\frac{1}{K}\overset{K}{\underset{k=1}{\sum }}p_{kij}^{U},\\ \;\begin{array}{cccc} \;C_{1} & C_{2} & \ldots & C_{n} \end{array}\\ \tilde{P}={\left({\tilde{p}}_{ij}\right)}_{\left[n\times n\right]}=\begin{array}{c} C_{1}\\ C_{2}\\ ...\\ C_{n} \end{array}\left[\begin{array}{cccc} 0 & {\tilde{p}}_{12} & \ldots & {\tilde{p}}_{1n}\\ {\tilde{p}}_{21} & 0 & \ldots & {\tilde{p}}_{2n}\\ \ldots & \ldots & {\tilde{p}}_{ij} & \ldots \\ {\tilde{p}}_{n1} & {\tilde{p}}_{n2} & \ldots & 0 \end{array}\right]. \end{array}$$
Step 2: The normalized direct-influence fuzzy matrix $\tilde{M}$ construction.
The elements ${\tilde{m}}_{ij}=\left(m_{ij}^{L},m_{ij}^{M},m_{ij}^{U}\right)$ in the normalized direct-influence fuzzy matrix $\tilde{M}$ can be calculated through the following equation:
  (6) $$\begin{array}{c} {\tilde{m}}_{ij}=\frac{{\tilde{p}}_{ij}}{s}=\left(\frac{p_{ij}^{L}}{s},\frac{p_{ij}^{M}}{s},\frac{p_{ij}^{U}}{s}\right)=\left(m_{ij}^{L},m_{ij}^{M},m_{ij}^{U}\right),\\ s=\underset{1\leq i\leq n}{\max}\left(\sum_{j=1}^{n}p_{ij}^{U}\right). \end{array}$$
Step 3: The development of the total-influence fuzzy matrix $\tilde{T}$.
The total-influence fuzzy matrix $\tilde{T}$ can be obtained from the following equation:
  (7) $$\begin{array}{c} \tilde{T}=\underset{k⟶\infty }{\lim}\left(\tilde{M}⊕{\tilde{M}}^{2}⊕\ldots ⊕{\tilde{M}}^{k}\right)=\tilde{M}{\left(I-\tilde{M}\right)}^{-1},\\ \tilde{T}={\left({\tilde{t}}_{ij}\right)}_{n\times n}, \end{array}$$
where ${\tilde{t}}_{ij}=\left(t_{ij}^{L},t_{ij}^{M},t_{ij}^{U}\right)$ and
  (8) $$\begin{array}{c} \left[t_{ij}^{L}\right]=M_{L}\times {\left(1-M_{L}\right)}^{-1},\\ \left[t_{ij}^{M}\right]=M_{M}\times {\left(1-M_{M}\right)}^{-1},\\ \left[t_{ij}^{U}\right]=M_{U}\times {\left(1-M_{U}\right)}^{-1}, \end{array}$$
where *I* is the *n* × *n* square matrix with ones on its diagonal.
Step 4: Establishment of criteria influential relation map.
The sum of rows and columns are obtained from the total-influence matrix respectively expressed as ${\tilde{D}}_{i}$ and ${\tilde{R}}_{i}$ equation (9). The criteria in effect group and cause group can be calculated based on the ordered pairs of (${\tilde{D}}_{i}+{\tilde{R}}_{i},{\tilde{D}}_{i}-{\tilde{R}}_{i}$).
  (9) $$\begin{array}{c} \tilde{D}={\left({\tilde{D}}_{i}\right)}_{n\times 1}={\left[\sum_{j=1}^{n}{\tilde{t}}_{ij}\right]}_{n\times 1},\tilde{R}={\left({\tilde{R}}_{j}\right)}_{1\times n}={\left[\sum_{i=1}^{n}{\tilde{t}}_{ij}\right]}_{1\times n}. \end{array}$$
According to equation (3), the fuzzy ordered pairs (${\tilde{D}}_{i}+{\tilde{R}}_{i},{\tilde{D}}_{i}-{\tilde{R}}_{i}$) are defuzzified to the crisp pairs (${\left({\tilde{D}}_{i}+{\tilde{R}}_{i}\right)}^{\text{def}},{\left({\tilde{D}}_{i}-{\tilde{R}}_{i}\right)}^{\text{def}}$) through GMIR method, as well as the elements in total-influence fuzzy matrix where ${\left({\tilde{D}}_{i}+{\tilde{R}}_{i}\right)}^{\text{def}}$ denotes the degree of the targeted attribute role that the factor plays in the network system and ${\left({\tilde{D}}_{i}-{\tilde{R}}_{i}\right)}^{\text{def}}$ means the net effect that the element contributes to the network system. In order to obtain the criteria influential relation map, the threshold value *p* is established based on total-influence matrix *T*. Only those influential relationships whose value is greater than the established threshold value should be kept and chosen in the CRM [73]. In this paper, the arithmetic mean of all elements in matrix *F* is *p* value [16]. If ${\left({\tilde{D}}_{i}-{\tilde{R}}_{i}\right)}^{\text{def}}>0$, it means the criterion *i* has an effect on other criteria which will belong to the *cause group*, and if ${\left({\tilde{D}}_{i}-{\tilde{R}}_{i}\right)}^{\text{def}}<0$, the attribute *i* is being affected by others, which will belong to the *effect group*.
Step 5: Subjective weight calculation.
Based on the following equation (10), the subjective weight of criteria can be obtained through CRM as **w**^*s*^=(*w*_1_^*s*^, *w*_2_^*s*^,…, *w*_*j*_^*s*^,…*w*_*n*_^*s*^).
  (10) $$\begin{array}{c} w_{i0}={\left({\left[{\left({\tilde{D}}_{i}+{\tilde{R}}_{i}\right)}^{\text{def}}\right]}^{2}+{\left[{\left({\tilde{D}}_{i}-{\tilde{R}}_{i}\right)}^{\text{def}}\right]}^{2}\right)}^{1/2};w_{i}^{s}=\frac{w_{i0}}{\sum_{i=1}^{n}w_{i0}}. \end{array}$$

### 3.3. Objective Weight by Antientropy Weight (AEW) Technique

Shannon Entropy is an effective method for uncertain information measurement formulated in terms of possibility theory. Liu has applied this technique into MCDM problem for the weights acquisition [74]. Objective weights based on entropy value can be realized through the following stages [75].

Step 1: Normalization of the decision-making matrix. The elements of the matrix can be calculated according to the following equation:
  (11) $$\begin{array}{c} {\text{P}}_{ij}=\frac{x_{ij}}{\sum_{i=1}^{m}x_{ij}}. \end{array}$$
Step 2: Calculation for the information entropy of each criterion based on the following equation:
  (12) $$\begin{array}{c} e_{j}=-k\sum_{i=1}^{m}p_{ij}lnp_{ij}=-\frac{1}{lnm}\sum_{i=1}^{m}p_{ij}lnp_{ij}. \end{array}$$
Step 3: The objective weight of each criterion can be obtained through the following equation:
  (13) $$\begin{array}{c} {\text{w}}_{j}^{o}=\frac{1-e_{j}}{\sum_{j=1}^{n}\left(1-e_{j}\right)}. \end{array}$$

### 3.4. Ranking Method Based on Fuzzy VIKOR Procedure

The VIKOR (VlseKriterijumska Optimizacija I Kompromisno Resenje) method has proven to be an effective method for multi-criteria prioritization problem [76–80]. The fuzzy VIKOR is the extension VIKOR method integrated with fuzzy-based techniques. The philosophy of VIKOR method is based on the particular measure of closeness to the ideal solution started with the following form of *L*_*p*_-metric.

(14) $$\begin{array}{c} L_{p,i}={\left\{{\sum_{j=1}^{n}\left[\frac{w_{i}\left(f_{j}^{*}-f_{ij}\right)}{f_{j}^{*}-f_{j}^{-}}\right]}^{p}\right\}}^{1/p},\;1\leq p\leq +\infty ,\;\;i=1,2,\ldots ,m. \end{array}$$

It can be ranked by the index to choose the compromise solution. The implementation steps of FVIKOR method are as follows [75]:

Step 1: The normalized difference d_*ij*_ calculation.
The normalized difference d_*ij*_ is calculated based on the best value *f*_*j*_^*∗*^ and worst value *f*_*j*_^−^ in following equation.
  (15) $$\begin{array}{c} {\text{d}}_{ij}=\frac{f_{j}^{*}-x_{ij}}{f_{j}^{*}-f_{j}^{-}}, \end{array}$$
where
  (16) $$\begin{array}{c} f_{j}^{*}=\left\{\begin{array}{c} \underset{i}{\max}x_{ij}\text{,the more the better},\\ \underset{i}{\min}x_{ij},\text{the less the better}, \end{array}\right.f_{j}^{-}=\left\{\begin{array}{c} \underset{i}{\min}x_{ij}\text{,the less the bad},\\ \underset{i}{\max}x_{ij},\text{the more the bad}. \end{array}\right. \end{array}$$
Step 2: Compute *S*_*i*_ and *R*_*i*_ with criteria combined weight
The relative importance of subjective weight compared with objectivity is *φ*. According to equations (10) and (13), the combined weight of criteria **w**^*c*^=(*w*_1_^*c*^, *w*_2_^*c*^, *w*_*j*_^*c*^,…, *w*_*n*_^*c*^) can be calculated. Then the maximum group utility value *S*_*i*_ and minimum individual regret value *R*_*i*_ can be obtained in equation.
  (17) $$\begin{array}{c} S_{i}=\sum_{j=1}^{n}\left(w_{j}^{c}\;{\text{d}}_{ij}\right),\\ R_{i}=\underset{j}{\max}\left(w_{j}^{c}\;{\text{d}}_{ij}\right),\\ w_{j}^{c}=\varphi w_{j}^{s}+\left(1-\varphi \right)w_{j}^{o}. \end{array}$$
Step 3: Calculation of the comprehensive utility value *Q*_*i*_,  *i*=1,2,…, *m*.
  (18) $$\begin{array}{c} Q_{i}=v\frac{S_{i}-S^{*}}{S^{-}-S^{*}}+\left(1-v\right)\frac{R_{i}-R^{*}}{R^{-}-R^{*}}, \end{array}$$
where $S^{-}=\underset{i}{\max}S_{i},S^{*}=\underset{i}{\min}S_{i},R^{-}=\underset{i}{\max}R_{i},R^{*}=\underset{i}{\min}R_{i}$. In order to reflect the attitude of decision makers, *vϵ*(0,1) represents the relative importance of maximum group utility, while the 1-*ν* is the relative importance of individual regret.
Step 4: Alternatives ranking based on the three index value: *S*, *R*, and *Q*. The candidate *A*^(1)^ will be regarded as the compromising solution, who has the minimum comprehensive group utility value *Q*, if the following two conditions (acceptance advantage and its stability) can be satisfied.

## 4. Case Study

### 4.1. Background and Data Collection

A real numerical case for the application of the hybrid MCDM approach integrating the fuzzy DEMATEL, anti-entropy method, and FVIKOR technique is presented in this section, and it has been applied into the quality cost framework selection of an automotive enterprise in China. The enterprise is a famous vehicle-assembly firm providing vehicle products such as cars, sport utility vehicles (SUVs), vans, and multipurpose vehicles (MPVs). With the implementation of quality improvement activities (8D and Six sigma), the quality index (PP100 and R/1000) is improved dramatically [67]. While, there is no appropriate quality cost framework helps managers to recognize the quality related cost and it is not enough to identify the COQ based on the financial report. In that case, it is of great urgency for CA Company to select the best quality cost framework to help its manager identify the COQ during the product whole lifecycle, especially for the continuous quality improvement procedure.

As the previous analyzed, there are four QCF alternatives in this study, which are evaluated from the two dimensions (effectiveness and feasibility). Expert panels include the quality manager, financial manager, and an expert on COQ. In order to obtain the required data, a questionnaire is prepared and distributed among the decision-making team, and each representative provide a judgment with linguistic variables for the direct influence of criteria (Table 6) and A1 alternative's performance subject to each criterion (Table 7), respectively.

In order to reflect the robustness of the proposed hybrid MCDM framework, the sensitivity analysis on the decision parameters *φ* and *v* are conducted in eleven experiment scenarios illustrated in Tables 8 and 9. In addition, in order to explore the best solution of the QCF under different consideration, the relative importance of the effectiveness (*ρ*) is defined with 11 experiment scenarios in Table 10.

### 4.2. Application of the Proposed Approach

The fuzzy DEMATEL method was used to recognize interdependence and influence relationships among the criteria. The initial fuzzy direct influence matrix provided by the three representatives was collected by pairwise comparison in terms of influences (Table 5) and the fuzzy average direct influence matrix $\tilde{P}$ was calculated based on equation (5). According to equations (6)–(9), the total-influence matrix $\tilde{T}$ was derived and the threshold value *p* is established. The various indexes calculation results by FDEMATEL method are presented in Table 11 and criteria relationship map (CRM) was drawn based on the order pairs ${\left({\tilde{D}}_{i}+{\tilde{R}}_{i}\right)}^{\text{def}},{\left({\tilde{D}}_{i}-{\tilde{R}}_{i}\right)}^{\text{def}}$, as shown in Figure 2. In addition, the objective weight of criteria based on AEW method based on equations (12)–(14) is illustrated in Table 11. Let *φ*  = 0.5, the combined weights can be calculated.

According to Table 11, the criteria weight can be obtained by fuzzy DEMATEL and antientropy method, which are embedded into fuzzy VIKOR procedures. The *S*, *R* and *Q* value and alternative ranking result can be obtained based on equations (15)–(18) as presented in Table 12.

As can be seen in the above table, the ranking order has the same sequence by *S*, *R,* and *Q* index. In addition, *Q*(*A*^(2)^) − *Q*(*A*^(1)^) = *Q*(*A*3) − *Q*(*A*4) = 0.42 ≥ *DQ* = 0.33. Therefore, the ABC quality cost framework (A4) is the best selection for its satisfaction on the two conditions. The research result shows high conformity with Tsai's study that the ABC model is the best choice for enterprise to recognize the economics of its quality improvement procedure [16]. Besides, the ranking lists show a high conformity with the TOPSIS-based method.

### 4.3. Sensitivity Analysis

The abovementioned analysis shows the application of the proposed hybrid MCDM approach for the quality cost framework selection. In order to analyze the robustness of the proposed method, the sensitivity analysis is performed to understand effect on ranking result of the decision parameters. Established experimental scenarios are set in Tables 8–10.

#### 4.3.1. Sensitivity Analysis on Relative Importance of Group Utility *v*

The relative importance of group utility *v* reflects the optimistic attitude, and the *Q* value reflects the comprehensive group utility of compromising solution. The calculated *Q* index values in different experimental scenarios (Table 8) are presented in the following Figure 3.

As Figure 3 shows, the best QCF selection is always the ABC model and the last one is PAF model (A1), even though there is a little fluctuation for the specific *Q* values of the middle two alternatives in different scenarios. The ranking order of the four quality cost framework alternatives keeps steady which means the group utility weight does not influence the decision result.

#### 4.3.2. Sensitivity Analysis on Relative Importance of Subjectivity *φ*

The defined decision parameter *φ* shows the relative importance of subjective weight, which reflects the weight of subjectivity in decision making. In this case, the sensitivity analysis on parameter *φ* (Table 9) is conducted to investigate the influence of subjectivity weight on the QCF alternative ranking results. The obtained *Q* values in established scenarios are illustrated in Figure 4.

The above figure shows high stability of the best solution (A4) when parameter *φ* varies. Similar to the sensitivity analysis result of parameter *v*, the *Q* value of the middle two alternatives in established 11 scenarios keep a slight fluctuation which does not influence the ranking order.

#### 4.3.3. Sensitivity Analysis on the Relative Importance of Effectiveness Dimension *ρ*

The decision parameter *ρ* reflects the attitude and validity of the representatives when the enterprise wants to select an appropriate quality cost framework. The conflict and paradox of the COQ model and traditional cost framework exist due to their unconformity. It is difficult for an organization to choose a best QCF with the two dimensions into consideration. In this part, the aim of sensitivity analysis is to explore the best solution variation when the firm focused on the different dimension.

As can be seen in the above Figure 5, the PAF quality cost framework is always the last alternative solution compared with other three ones. While the *Q* index values and ranking orders of other three alternatives fluctuate dramatically. When *ρ*≤ 0.5, the organization focuses on the feasibility of quality cost framework, and the best solution is ABC model catered to Tsai's research. However, when *ρ* > 0.5, the intangible loss quality cost framework shows its priority than other three alternatives due to the dominance of effectiveness dimension of QCF.

### 4.4. Discussion and Management Insight

The sensitivity analysis on the three decision parameters has been conducted to analyze the robustness of the proposed hybrid MCDM method. The analysis result shows that the best solution keeps a stable priority in terms of parameter *v* or *φ*. However, best selection shifts from A4 to A2 with the increasing of parameter *ρ*. It is very interesting to find the different research conclusion compared with Tsai's research that the ABC model priors to other alternatives when the organization focuses on the feasibility of quality cost framework, while the intangible cost model shows its priority when it concentrates on effectiveness dimension. When the CA organization focus on the effectiveness dimension of quality cost framework, the intangible cost framework is more appropriate.

The best solution change means Chinese companies tend to focus on the importance of the hidden cost due to product unconformity, customer complaints and reputation loss, since they want to take these intangible cost items into consideration in its quality cost framework and costing report. However, it is really very difficult to quantify the cost item for either PAF model or intangible cost framework for manufacturing firms. Even some published papers have been studied on the quality cost calculation, the specific application was usually based on the organization's particular requirement. The QCF selection is a team task with all related departments involvement, and this paper presented a systematic procedure to establish an appropriate QCF integrating decision information from multigroups. The manager can select the appropriate quality cost framework based on the practical consideration of the organization. Actually, as Schiffauerova and Thomson studied [11], the quality cost framework alternative is only just a basic concept and the concrete costing systems or costing report still differ from company to company.

From the case application of the investigated organization in this paper, there occur two kinds of best solution, one is the ABC model and the other is the intangible loss framework. The intangible loss quality cost framework is the best choice when decision makers pay more attention on effectiveness principle and it can illustrate the quality related cost item from prevention, appraisal and failure term, as well as the hidden cost, which provides and extensive looking. While the best choice is the activity-oriented cost (ABC) measurement method when decision makers focus on feasibility dimension more, and it can help manager to investigate specific cost item. The new quality cost framework from lifecycle and COQ dimension would be welcomed for both effectiveness and feasibility.

## 5. Conclusions

This paper employed a hybrid fuzzy multicriteria approach for quality cost framework selection from the typical four alternatives (PAF, intangible cost, process cost, and ABC), which helps the quality manager to develop quality cost practice based on appropriate QCF. The case study by the hybrid fuzzy MCDM approach integrating fuzzy DEMATEL, anti-entropy weighting technique, and fuzzy VIKOR method shows high robustness and flexibility on decision parameters. In addition, the fuzzy-based technique has been adopted to facilitate the decision makers to collect decision information. According to the model result, it caters to Tsai's study when the organization concentrates on feasibility principle, while the intangible loss cost framework shows the top priority when decision makers pay more attention to effectiveness for CA organization. This hybrid fuzzy MCDM approach shows its advantage on the flexibility of decision making and easy implementation due to the combined weighting technique and fuzzy method, and the auto-factory can perform quality costing practice based on this selection model. However, this study carries some limitations. First, the influential criteria can be extended based on different organizational industries by considering specific characteristics of individual requirements. Second, the decision-making information mainly comes from the judgements of experienced expert panels, and the big data driven techniques can be developed to make full use of operational information of objective firms. Finally, the AI-based decision-making framework could be explored to achieve smart determination and reduce the subjectivity.

## Figures and Tables

**Figure 1:** Membership function of triangular fuzzy number (TFN).

**Figure 2:** Criteria relationship map (CRM) in the two dimension clusters.

**Figure 3:** Sensitivity analysis on group utility weight *v*.

**Figure 4:** Sensitivity analysis on importance of subjective weight *φ*.

**Figure 5:** Sensitivity analysis on relative importance of two principles *ρ*.

**Table 1:** Four typical quality cost framework details.

	Prevailing QCF	Details and cost items	References
A1	PAF framework	Prevention + appraisal + failure cost	[35–40]
A2	Intangible loss framework	Prevention + appraisal + failure + hidden cost	[29, 41–45]
A3	Process framework	Conformance + non-conformance cost	[19, 28, 46]
A4	ABC framework	Value-added + non-value-added cost	[30, 37, 47]

**Table 2:** General quality cost items by various nations.

Nations	QCF category	QCF items
ASQC (US)	A1-PAF	Prevention + appraisal + failure
BS6143 (UK)	A3-process cost	Conformance and non-conformance
ISO9004-1	A1-PAF	Prevention + appraisal + failure
GB/T13339 (CN)	A2-IL	Prevention + appraisal + internal/external failure

**Table 3:** Specific criteria for the requirement of a beneficial COQ framework.

Dimension	Criteria	Detail description
D1-effectiveness	C1	The selected alternative should support the continuous quality improvement procedures (CQIP)
	C2	The selected alternative should contain as many COQ items as possible
	C3	The selected alternative should be applicable to all the departments of the organizations

D2-feasibility	C4	The selected alternative should have an easy data collection and application
	C5	The selected alternative should have the clear form and type of data needed
	C6	The selected alternative should be based on the concept of production procedures
	C7	The cost item of selected alternative should be easily recognized, calculated and recorded by the organization

**Table 4:** Linguistic variables and corresponding TFNs for criteria influence degree.

Linguistic variables of influence description	Triangular fuzzy number (TFN)
No influence (NI)	(0, 0, 0.25)
Very low influence (VL)	(0, 0.25, 0.5)
Low influence (L)	(0.25, 0.5, 0.75)
High influence (HL)	(0.5, 0.75, 1)
Very high influence (VH)	(0.75, 1, 1)

Source: [59–61].

**Table 5:** Linguistic variables and corresponding TFNs for alternative evaluation.

Linguistic variables of influence description	Triangular fuzzy number (TFN)
Very low/poor (VL/VP)	(0, 0, 0.25)
Low/poor (L/P)	(0, 0.25, 0.5)
Medium (M)	(0.25, 0.5, 0.75)
High/good (H/G)	(0.5, 0.75, 1)
Very high/good (VH/VG)	(0.75, 1, 1)

Source: [69].

**Table 6:** Initial direct influence degree of criteria given by representatives.

Effectiveness		C1	C2	C3	
C1	DM1	NI	VL	NI	
	DM2	NI	L	VL	
	DM3	NI	VL	VL	

C2	DM1	VH	NI	VH	
	DM2	HL	NI	VH	
	DM3	HL	NI	HL	

C3	DM1	VH	L	NI	
	DM2	L	VL	NI	
	DM3	VH	NI	NI	

Feasibility		C4	C5	C6	C7

C4	DM1	NI	VL	NI	L
	DM2	NI	L	VL	VL
	DM3	NI	L	VL	HL

C5	DM1	HL	NI	L	HL
	DM2	VH	NI	VL	VH
	DM3	VH	NI	NI	L

C6	DM1	HL	VL	NI	NI
	DM2	L	VL	NI	NI
	DM3	VH	NI	NI	VL

C7	DM1	HL	L	VL	NI
	DM2	VH	L	HL	NI
	DM3	VH	HL	L	NI

**Table 7:** Linguistic ratings of A1 QCF subject to criteria.

		C1	C2	C3	C4	C5	C6	C7
A1-PAF	DM1	G	M	VP	M	P	VP	P
	DM2	M	P	VP	P	M	G	M
	DM3	P	G	M	VP	P	P	VP

**Table 8:** Group utility weight setting (11 scenarios).

	SA1	SA2	SA3	SA4	SA5	SA6	SA7	SA8	SA9	SA10	SA11
*v*	0	0.1	0.2	0.3	0.4	0.5	0.6	0.7	0.8	0.9	1

**Table 9:** Relative importance of subjective weight (11 scenarios).

	SB1	SB2	SB3	SB4	SB5	SB6	SB7	SB8	SB9	SB10	SB11
*φ*	0	0.1	0.2	0.3	0.4	0.5	0.6	0.7	0.8	0.9	1

**Table 10:** Relative importance of “effectiveness” compared with feasibility principle (11 scenarios).

	SC1	SC2	SC3	SC4	SC5	SC6	SC7	SC8	SC9	SC10	SC11
*ρ*	0	0.1	0.2	0.3	0.4	0.5	0.6	0.7	0.8	0.9	1

**Table 11:** Criteria weight item calculation result.

	$\left({\tilde{D}}_{i}+{\tilde{R}}_{i}\right)$	$\left({\tilde{D}}_{i}-{\tilde{R}}_{i}\right)$	Group	*w*_*j*_^*s*^	*w*_*j*_^*o*^	*w*_*j*_^*c*^

C1	(0.631, 1.267, 3.750)	(−1.371, −0.569, −0.514)	Effect	0.099	0.140	0.119
C2	(0.780, 1.861, 6.388)	(0.561, 0.772, 1.337)	Cause	0.148	0.161	0.153
C3	(0.665, 1.709, 6.027)	(−0.117, −0.051, 0.008)	Effect	0.129	0.109	0.119
C4	(1.010, 2.352, 9.064)	(−1.490, −0.780, −0.567)	Effect	0.193	0.117	0.155
C5	(0.680, 1.791, 7.913)	(0.121, 0.131, 0.169)	Cause	0.151	0.156	0.153
C6	(0.327, 1.170, 6.472)	(0.103, 0.140, 0.249)	Cause	0.110	0.159	0.134
C7	(0.830, 2.039, 8.548)	(0.294, 0.509, 1.120)	Cause	0.171	0.158	0.164

**Table 12:** Four QCF alternatives ranking result based on *S*, *R* and *Q* value.

*Alternative*	The proposed integrated framework				TOPSIS-based method	
	*S* value	*R* value	*Q* value	Ranking by *S*/*R*/*Q*	*RC value by the TOPSIS steps*	Ranking by *RC*
A1-PAFF	0.892	0.164	1	4	0.492	4
A2-ILF	0.513	0.155	0.563	3	0.523	3
A3-PF	0.370	0.153	0.420	2	0.758	2
A4-ABCF	0.319	0.119	0	1	0.952	1

## Data Availability

The data used to support the findings of this study are included within the article.
